This article has been retracted.

# A Clinical Study on the Brain Protection Effect of Propofol Anesthesia on Patients Undergoing Acute Craniocerebral Trauma Surgery Based on Blockchain

**DOI:** 10.1155/2022/6111543

**Published:** 2022-04-09

**Authors:** Hu Li, Jinfeng Li, Peng Su, JianJun Zhang, Ding Ma

**Affiliations:** ^1^Department of Anesthesiology, Sichuan Academy of Medical Sciences & Sichuan Provincial People's Hospital, Chengdu 610032, China; ^2^Department of Anesthesiology, Chengdu Seventh People's Hospital, Chengdu 610041, China

## Abstract

In order to explore the effects of propofol anesthesia system based on block chain on brain tissue and brain function protection, 88 patients undergoing craniocerebral trauma surgery are selected for prospective study. The anesthetic dose of propofol during operation in the control group is determined according to general information and personal situation. The team uses blockchain to process the patient's clinical data and general information to calculate the optimal dose of propofol. The changes of hemodynamic indexes of patients in the two groups are compared, including dural incision (T1), 1 h after craniotomy (T2), end of surgery (T3), and 6 h after surgery (T4). The changes of neuron-specific enolase (NSE) and central neuron-specific protein (S100*β*) at T1, T2, T3, and T4 in 2 groups are observed and recorded. The changes of malondialdehyde (MDA) at T1, T2, T3, and T4 are compared between the two groups. Based on the analysis of clinical data and general information of patients on blockchain, the optimal intraoperative anesthetic dose of propofol for patients can effectively protect the brain function of patients, and the intraoperative anesthesia state is relatively stable, and the changes and improvements of intraoperative indicators are good.

## 1. Introduction

As a special term in the field of information technology, blockchain, as the data and information stored in a shared database, has the characteristics of open and traceable source and cannot be forged. Therefore, blockchain technology is gradually applied in a variety of fields and has laid a solid foundation for trust and cooperation [1, 2]. According to the study, one of the challenges faced by the healthcare industry includes medical data sharing. Traditional way case save cases in paper and electronic medical records, and the paper case has the characteristics of easy to loss, easy to damage, and the save time is shorter. Electronic medical record's intact degree is higher, but the hospital network system security may be poor and vulnerable to hacker attacks and may involve dereliction of duty of the medical staff or accidental disclosure of patients' medical records, posing a threat to patients' personal property and information [3, 4]. In addition to the inability to share traditional medical data, it may also lead to poor treatment outcomes or delays in treatment. Therefore, the exchange and sharing of medical data can not only ensure the privacy of patients but also solve the problem of lack of medical information [5].

Acute craniocerebral trauma refers to cerebral vascular rupture and hemorrhage and brain tissue damage caused by fall or impact. It has the characteristics of high mortality and rapid progress and is also one of the common diseases in neurosurgery. At present, the treatment of craniocerebral trauma is mainly surgery, but surgery is traumatic treatment, so the brain function and brain tissue will have a certain impact, so the choice of narcotic drugs is particularly important [6]. Studies have shown that propofol, as an anesthetic for preoperative induction and maintenance, can maintain the balance of cerebral oxygen supply and demand, thus playing a role in brain protection and can reduce the level of oxygen free radicals in patients with head trauma, thus reducing brain injury, with good clinical efficacy [7, 8]. However, in the present clinical use of propofol in patients with craniocerebral trauma with most of the patient's general information and doctor's clinical experience, the lack of the previous medical data makes the doctor cannot combine the patient information for fine adjustment of the dose of propofol, resulting in some patients to regain consciousness with extension or no ideal improvement in indicators and cannot achieve the expected goal [9–12]. Therefore, this study establishes a medical data system based on blockchain so as to determine the anesthetic dose of propofol in detail and observe the changes of perioperative indicators related to brain function in patients with head trauma so as to explore the clinical feasibility of this scheme [13–15]. It will be reported as follows.

## 2. General Patient Information and Methods

### 2.1. General Patient Information

The patients were selected from January 2020 to January 2021. Our prospective study involves 88 cases of patients with craniocerebral trauma surgery. According to patients' personal wishes, they were divided into control group (*n* = 45) and study group (*n* = 43). The control group patients were treated in accordance with the general information and determined the propofol dosage based on doctor's clinical experience. The study group patients were treated through building blockchain system of medical data. The dosage of propofol is determined after analysis [16–18]. There are 21 males and 24 females in the control group, aged 52–64 years, with an average of (58.23 ± 5.62) years. There are 25 males and 18 females in the study group, aged 53–63 years, with an average of (57.23 ± 5.38) years. There is no significant difference in general data between the two groups (*P* > 0.05), indicating comparability. All patients included in this study signed informed consent and are grouped according to the wishes of individuals or their families. The clinical data and general information are kept confidential and used for research purposes only, not other purposes. Inclusion criteria are as follows: (1) no serious kidney injury; (2) all signed informed consent; (3) meet the diagnostic criteria of acute craniocerebral trauma; and (4) no respiratory tract infection. Exclusion criteria are as follows: (1) respiratory arrest before surgery; (2) poor compliance of family members and patients, unable to cooperate with the study; (3) people with a history of allergy to propofol; and (4) lack of clinical data.

### 2.2. Methods

The construction of blockchain medical data, anesthesia operation, and index detection methods in this study are described as follows.

#### 2.2.1. Establishment of Blockchain Medical Data

1. For patients with previous medical records, it could provide complete medical information to patients as much as possible through oral inquiry. At the same time, doctors can change the right of patients to obtain medical information according to the change confirmation of patients' medical information, so the future medical disputes can be traced back to the source.
2. The medical information of patients was encrypted through the hash algorithm, and the medical data of patients is treated as block information and compressed into strings, which can only be parsed through a unique hash algorithm to ensure data security.
3. The medical data established by blockchain was treated as a third-party platform, and the block chain technology was used to export specific hash values so that hospitals, patients, and regulatory sites can obtain the hash values through legal ways, and read the data and also play a role of mutual supervision.
4. After the blockchain medical data system is completed, it can be divided into two modules and medical record management. First of all, for all patients who visit for the first time, they could use ID and name to enter the system. At the end of the visit, the outpatient information recorded and stored in the node will be uploaded automatically. When the patient visits again, the doctor will be authorized to query the records and drugs. Detailed diagnosis is performed.

#### 2.2.2. Anesthesia Operation

Patients in both groups are treated with tracheal intubation for general anesthesia, anesthesia induction is performed with 1 mg/kg lidocaine, 0.1 mg/kg vecuronium, and 2 *µ*g/kg fentanyl, and anesthesia maintenance is performed with propofol during surgery. The dosage of propofol is intravenous infusion according to the preoperative dose of clinical data analysis of patients in both groups.

#### 2.2.3. Hemodynamic Detection

5 ml of patients' venous blood is taken at T1, T2, T3, and T4 and centrifuged at 3000 r/min for 5 min. After centrifugation, the upper serum is taken and stored in a refrigerator at −70°C for later use. Preoperative and postoperative mean arterial pressure (MAP) is monitored by arterial pressure detector. Patients' heart rate (HR) is monitored using 24-hour ambulatory electrocardiogram.

#### 2.2.4. Determination Methods of Other Indicators

The serum neuron-specific enolase (NSE) is determined by the chemiluminescence method with an imported automatic electrochemiluminescence instrument. The content of central nervous specific protein (S100*β*) is determined by double antibody sandwich ELISA. The concentration of malondialdehyde (MDA) is measured with the thiobarbituric acid colorimetric method.

All the data in this study are collected and sorted out, and put into SPSS23.0 for statistical data processing. The measurement data are expressed as ($\bar{x}$ ± *S*), and intergroup differences are performed by independent sample *t*-test, intragroup comparison by paired *t*-test, and intergroup comparison by the F test. Repeated measurement ANOVA is used to perform the spherical test among multiple groups. Count data are represented by (%), and differences between groups are tested by *χ*^2^. When *P* < 0.05, the difference between data is statistically significant.

## 3. The Experimental Results

### 3.1. Comparison of Changes in Hemodynamic Indexes at Different Time Periods

There is no statistical significance in HR between the two groups (*P* > 0.05), and MAP showed no significant difference at T1 and T2 but changed in T3 and T4. The study group is more stable than the control group (all *P* < 0.05), as shown in Table 1. Table 1 shows changes of hemodynamic indexes.  Figure 1 shows the comparison of changes in hemodynamic indexes at different time periods.

### 3.2. Comparison of changes of NSE and S100*β* at Different Time Periods

T1 and T2 NSE had no significant differences found. The level of NSE in T3 and T4 groups is increased, but that in the study group is significantly lower than that in the control group (*P* < 0.05). Meanwhile, S100*β* showed an upward trend in both groups. The level of S100*β* in the study group is lower than that in the control group at T3 and T4 time points (*P* < 0.05), as shown in Table 2.  Figure 2 displays the comparison of changes of NSE and S100*β* in different time periods.

### 3.3. Comparison of MDA Index Changes at Different Time Points

The MDA level in the study group is lower than that in the control group at T3 and T4 time points, and the MDA level in both groups showed a downward trend (*P* < 0.05), as shown in Table 3.  Figure 3 presents the comparison of MDA index changes at different time points.

## 4. Experimental Result Analysis

Medical information is a patient's disease data. The more complete the medical information is, the more doctors can prepare to judge the condition and make targeted plans. Especially for patients with complex or complicated diseases, a safe and complete medical record is more efficient to evaluate the condition. Now in the process of the patient's disease diagnosis, clinicians often diagnose through oral questioning of the patient's medical history. This method has many disadvantages, such as when a patient is unable to accurately remember past disease specific values, nonmedical proper nouns in the described condition at the same time also can affect the judgment of the condition by the doctor. In order to solve this situation, many medical institutions keep medical records in a computer system so that patients can refer to it for reference in the next visit. However, if patients seek treatment in different hospitals or different departments in the same hospital, there will be many obstacles in the implementation of this method. With the continuous development of computer science, the concept of blockchain is gradually applied to medical data storage. By forming distributed ledger on computer nodes, it can not only solve the problem of medical information being easy to be tampered with, but also solve the problem of medical information island through data sharing across the board. Some scholars pointed out that in craniocerebral trauma surgery, anesthesia, as one of the most important steps in the process of operation, and its dosage or improper operation is easy to damage the patient's brain function. However, because of the lack of medical information, some error occurs on preoperative anesthesia evaluation, causing coma after surgery in patients with prolonged drop of cerebral oxygen supply. Therefore, it is of great significance to share the medical information of patients with head trauma and apply it in propofol anesthesia. However, at present, there is no relevant study on propofol anesthesia applied by blockchain at home and abroad. Therefore, the most appropriate anesthetic dose of propofol was constructed by blockchain, and a prospective study was conducted to explore the influence of the estimated dose of propofol after blockchain data sharing on the postoperative brain protection of patients with acute craniocerebral trauma.

According to the results of two groups of patients with changes in the levels of MAP in T1, T2 is not significant. In T3 and T4, it is decreased and relatively stable (*P* < 0.05), prompted after building blockchain of propofol anesthesia and can better maintain hemodynamic stability, avoid index's volatility, and effectively maintain intraoperative postoperative blood circulation stability. However, HR detection found that there is no significant difference in heart rate changes in the four periods, so there is little influence on the heart rate. As one of the enolase involved in the glycolysis pathway, NSE is widely distributed in nerve and neuroendocrine tissues and expresses the highest activity in brain tissues. As a molecular marker with high clinical application value, NSE is often used to detect neuroblastoma and small cell lung cancer. It is also one of the important indicators often used to judge whether the brain is protected or not in clinic. When brain neurons are damaged, NSE will flow out of neurons into the blood, leading to an increase in serum detectable NSE level. Therefore, the higher the level of NSE, the more serious the brain injury degree of the patient. In this study, the level of NSE in both groups increased after craniotomy, but the level of NSE in the study group is significantly lower than that in the control group (*P* < 0.05), indicating that propofol anesthesia constructed based on blockchain has a certain effect on brain protection. In addition, S100*β* protein, as the “C-reactive protein” in the brain, is stored in the central nervous system in large quantity. It has a wide range of biological activities and can mediate cell proliferation, differentiation, and apoptosis. When patients with brain injury, S100*β* will infiltrate into the cerebrospinal fluid from nerve cells and enter the blood through the damaged blood-brain barrier, resulting in the increase of serum S100*β* concentration. Bersani I indicated that S100*β* has a high clinical value in the diagnosis and prognosis of brain injury. The higher the serum concentration of S100*β*, the more severe the brain injury and the worse the prognosis, and the trend increased with the aggravation of the disease. In this study, the level of S100*β* increased in both groups after craniotomy, but the concentration of S100*β* in the study group is lower than that in the control group (*P* < 0.05), indicating that propofol anesthesia based on blockchain has a good protective effect on brain. As the final product of lipid peroxidation reaction in the body, MDA can induce the polymerization of proteins, nucleic acids, and other molecules, causing cytotoxicity, and the generation of MDA can aggravate membrane damage. Therefore, the determination of serum MDA can not only reflect the degree of lipid peroxidation in the body, but also reflect the degree of brain cell damage. The results of this study showed a downward trend in MDA levels in both groups, but lower in the study group (*P* < 0.05), suggesting that propofol anesthesia based on blockchain can reduce the MDA output, thus playing a role in brain protection.

## 5. Conclusion

In conclusion, the propofol anesthesia system based on the analysis of medical data based on blockchain can maintain the stability of patients' hemodynamics during and after surgery as well as the effect of brain protection, so it has good clinical application value.

Although some achievements have been made in this study, there are still many shortcomings. First, the sample size selected in this study is small, and there are many differences among people in different countries and regions. Therefore, the sample size should be further expanded in the next study to make the research results more representative. Secondly, there are few studies on the application of blockchain in propofol anesthesia at home and abroad, and no scholars have demonstrated it yet. Therefore, the conclusions obtained in this study need to be further explored in the future, in order to lay a theoretical foundation for better protection of brain function in patients with acute craniocerebral trauma.

## Figures and Tables

**Figure 1:** Comparison of changes in hemodynamic indexes at different time periods.

**Figure 2:** Comparison of changes of NSE and S100*β* in different time periods.

**Figure 3:** Comparison of MDA index changes at different time points.

**Table 1:** Changes of hemodynamic indexes.

	Control group (*n* = 45)	Study group (*n* = 43)	*t*	*P* value
MAP (mmHG)				
T1	95.21 ± 11.23	96.24 ± 12.36	−0.409	0.683
T2	94.52 ± 12.31	93.52 ± 10.32	0.412	0.681
T3	90.21 ± 11.32^*∗*^	85.42 ± 10.43^*∗*^	2.062	0.042
T4	90.29 ± 10.27^*∗*^	84.46 ± 12.09^*∗*^	2.442	0.017
*F*	5.241	3.313		
*P* value	0.423	＜0.001		

HR (time/min)				
T1	79.42 ± 9.32	80.21 ± 9.62	−0.391	0.697
T2	76.24 ± 9.36	78.31 ± 9.24	−1.044	0.300
T3	77.24 ± 9.17	76.36 ± 9.54	0.441	0.660
T4	76.24 ± 9.52	78.52 ± 9.27	−1.138	0.258
*F*	4.257	5.863		
*P* value	0.291	0.128		

^*∗*^Changes of T3 and T4 indicators are statistically significant compared with T1.

**Table 2:** Changes of NSE and S100*β* indexes.

	Control group (*n* = 45)	Study group (*n* = 43)	*t*	*P* value
NSE （ng/ml）				
T1	2.94 ± 0.41	2.91 ± 0.42	0.339	0.735
T2	2.74 ± 0.56	2.78 ± 0.42	−0.378	0.707
T3	4.67 ± 1.02^*∗*^	4.01 ± 1.04^*∗*^	3.005	0.003
T4	5.85 ± 1.27^*∗*^	4.72 ± 0.52^*∗*^	5.416	＜0.001
F	5.241	3.313		
*P* value	＜0.001	＜0.001		

s100*β* (mmol/L)				
T1	1.23 ± 0.12	1.22 ± 0.19	0.297	0.767
T2	1.32 ± 0.34^*∗*^	1.36 ± 0.24^*∗*^	*P* < 0.050.635	0.527
T3	1.92 ± 0.41^*∗*^	1.45 ± 0.42^*∗*^	5.312	＜0.001
T4	2.68 ± 0.61^*∗*^	1.58 ± 0.73^*∗*^	7.684	＜0.001
F	4.257	5.863		
*P* value	＜0.001	＜0.001		

^*∗*^Changes of T2, T3, and T4 indicators are statistically significant compared with T1.

**Table 3:** Changes of MDA.

	Control group (*n* = 45)	Study group (*n* = 43)	*t*	*P* value
MDA (U/L)				
T1	57.24 ± 10.53	57.32 ± 10.42	−0.036	0.972
T2	56.31 ± 10.25	54.21 ± 11.27	0.915	0.363
T3	52.25 ± 9.46^*∗*^	46.63 ± 10.24^*∗*^	2.676	0.009
T4	50.58 ± 10.23^*∗*^	43.13 ± 9.12^*∗*^	3.600	0.001
*F*	5.241	3.313		
*P* value	＜0.001	＜0.001		

^*∗*^Compared with T1, the changes of T3 and T3 indicators are statistically significant.

## Data Availability

The simulation experiment data used to support the findings of this study are available from the corresponding author upon request.
